# Social Recommendation System Based on Hypergraph Attention Network

**DOI:** 10.1155/2021/7716214

**Published:** 2021-11-05

**Authors:** Zhongxiu Xia, Weiyu Zhang, Ziqiang Weng

**Affiliations:** School of Computer Science and Technology, Qilu University of Technology (Shandong Academy of Sciences), Jinan, Shandong 250353, China

## Abstract

In recent years, due to the rise of online social platforms, social networks have more and more influence on our daily life, and social recommendation system has become one of the important research directions of recommendation system research. Because the graph structure in social networks and graph neural networks has strong representation capabilities, the application of graph neural networks in social recommendation systems has become more and more extensive, and it has also shown good results. Although graph neural networks have been successfully applied in social recommendation systems, their performance may still be limited in practical applications. The main reason is that they can only take advantage of pairs of user relations but cannot capture the higher-order relations between users. We propose a model that applies the hypergraph attention network to the social recommendation system (HASRE) to solve this problem. Specifically, we take the hypergraph's ability to model high-order relations to capture high-order relations between users. However, because the influence of the users' friends is different, we use the graph attention mechanism to capture the users' attention to different friends and adaptively model selection information for the user. In order to verify the performance of the recommendation system, this paper carries out analysis experiments on three data sets related to the recommendation system. The experimental results show that HASRE outperforms the state-of-the-art method and can effectively improve the accuracy of recommendation.

## 1. Introduction

With the prosperity and development of social media, social networking sites have become an indispensable part of people's daily life. On these social media platforms, users can view or publish information and strengthen their connection with friends in life [1]. In addition, the behavior information of friends will also affect the attitude and behavior of a user, which we call social influence [2]. In order to help users discover potential attention information, social media platforms will also recommend the content of interest to users, which helps users to establish connections with other people who have similar interests. This behavior of users is called homophily [3]. The establishment of a social recommendation system is very important for the operation and development of social networking sites. Generally speaking, when a new user signs up to a new website, his friends help the platform recommend new items for him, which effectively solves the cold start problem [4]. If user-item interaction data is sparse, the recommendation system can infer the user's interests according to the interaction between users and friends, which alleviates the problem of data sparsity to a certain extent [5, 6], so as to better generate the recommended content for the user. Because the social recommendation system shows better performance than the general recommendation system [7, 8], it has attracted more and more attention from researchers.

In recent years, with the development of deep learning technology, graph neural networks (GNNs) [9] have been widely used in various fields of artificial intelligence. GNNs are highly valued in the field of social recommendation because of their powerful ability to fit graph data [10–13]. Different from the traditional social recommendation method based on deep learning, the method based on GNNs abstracts the data based on social relations into graph data and models the relation between users as pairwise relations, which helps the model to accurately learn the feature vectors of users. However, compared with traditional deep learning methods, existing models are not effective enough. The reason is probably that they ignore the higher-order relations among users. The high-order relation between users is relative to the first-order relation between users. The first-order relation between users refers to the paired user relations, while the high-order relation between users refers to multiple neighbor nodes related to user nodes. For example, two or more users are friends with each other or strangers who have similar interests with the users. We call these relations high-order relations between users (as shown in Figure 1). Obviously, there are complex high-order relations between users, and simple graphs cannot describe such high-order relations. Therefore, GNNs-based social recommendation methods cannot capture such complex high-order user relations.

In order to solve the above problem, we propose a new social recommendation method based on a hypergraph to model the high-order relations between users in social networks. Conceptually, hypergraph [14] makes up for the defect that traditional graphs can only connect pairs of nodes. That is, each edge in a hypergraph can connect multiple nodes. This structure supports the capture of complex high-order relations between users. The advantage of hypergraph modeling is that it can fully mine the relations between various users, thus avoiding the loss of information. Technically, we model complex high-order relations between users as nodes of specific triangular relations to construct hypergraphs, and these triangular relations are used to describe different semantic topics (as shown in Figure 1). These types of graphs embody different high-order relations between users, including “having common friends,” “friends buying the same item together,” and “strangers buying the same item”.

However, some node information is very important when propagating and aggregating user intentions within the hypergraph of triangular semantic topics, while others are not. In addition, for user nodes, there are different degrees of influence among users. Therefore, a key challenge is how to highlight the nodes with important information on each hyperedge. To meet this challenge, this paper proposes a model of applying a hypergraph attention network to social recommendation system (HASRE) by integrating hypergraph and graph attention network (GAT) [15]. In this model, the hypergraph is constructed to learn user information with high-order relations. At the same time, its internal exploit graph attention mechanism can learn key user information in the hypergraph. Finally, the user information with high-order relation information is combined with other user information obtained through graph convolution neural network (GCN) [16] to obtain a comprehensive user representation. Finally, combined with item embedding, the recommendation performance can be significantly improved.

Our contribution can be summarized as follows:

1. In this paper, the hypergraph model is used to model the relation between users, which can better capture the high-order user relation
2. We creatively incorporate the graph attention network into the hypergraph structure, which can pay more attention to the information of important users
3. We carry out analysis experiments on three data sets related to the recommendation system and finally proved that the model in this paper is superior to other state-of-the-art recommendation methods

## 2. Related Work

### 2.1. Recommender Systems

With the development of the Internet, recommendation systems achieved success in many fields, including e-commerce [17], social network [18], medical care [19], and other fields. Recommendation systems can help users find useful information in the huge amount of information and recommend items of interest to users. Because of these advantages, it has been favored by researchers in industry and academia [20, 21]. With the continuous improvement of computer algorithms, the development of the recommendation system is mainly divided into two stages: the traditional recommendation system and the deep learning-based recommendation system. The traditional recommendation systems are mainly divided into three categories. The content-based recommendation method mainly obtains the items that users are interested in from the interactive information between users and items and then recommends similar items for users [22]. The collaborative filtering recommendation method is the most widely used technology in the field of recommendation systems. It collects a large amount of information of users, mines the potential needs of users according to this information, and plays an auxiliary role in users' decisions [23]. The hybrid recommendation method combines the first two recommendation methods, which can better improve the performance of recommendation systems. The recommendation method based on deep learning is to apply the deep learning technology to the recommendation system, which can directly extract more useful information from user-item interaction information, so as to improve user satisfaction [24, 25]. Although there is still a certain gap between the item recommended by the system and people's needs, recommendation systems still play an important role in practical applications and provide a great convenience for people's life.

### 2.2. Graph Neural Network in Recommender Systems

In recent years, Graph Neural Network (GNN) [9] has attracted more and more attention and has brought great improvement in the fields of computer vision and natural language processing [26]. Because GNNs can effectively learn complex graph data, researchers have tried to apply graph neural network technology to the recommendation system, trying to improve the performance of the recommendation system, and achieved success. GC-MC [27] is a graph automatic encoder framework for matrix completion tasks in recommendation systems, which includes auxiliary information for users and items. PinSage [28] effectively combines random walk and graph convolution neural networks to capture the characteristics of graph structure and nodes to generate the embedded representation of nodes. These representative works all show that the application of GNNs to the traditional recommendation system can improve the performance of recommendations.

Since social networks can be seen as user-user interaction graph, it is natural to apply GNNs to social recommendations. SocialGCN [10] combines the advantages of GCNs in modeling diffusion processes in social networks with classical models based on potential factors to capture users' preferences. DiffNet++ [11] models influence diffusion and interest diffusion of neural networks in a unified framework based on DiffNet [12]. DICER [13] uses a perceptual graph neural network to learn the feature information of the graph and extract relevant information from deep context. Although these works are effective, these models are limited by the traditional graph structure, which can only use paired user relations and cannot capture the high-order relations of users, which leads to poor performance of the recommendation system.

### 2.3. Hypergraph in Recommender Systems

Hypergraph makes up for the defects of traditional graph structure, and it can model the high-order information of data [29]. With the rise of GNNs, hypergraph neural network has attracted more and more attention. HGNN [30] uses hyperedge convolution operation to deal with complex and high-order relational data, which is the earliest research work that combines graph convolution networks with a hypergraph. Based on the hyperedge convolution neural network (HGCN) [31], DHGNN [32] dynamically integrates feature embedding into hypergraph structure, thus obtaining local and global relations of data. Zhang et al. [33] applied an attention mechanism on hypergraphs to deal with hyperedge structures of different sizes. In recent years, hypergraph neural networks have achieved success in computer vision [34, 35], financial forecasting [36], natural language processing [37], and other fields.

Although hypergraph neural network shows the potential of high-order relational modeling in many fields, there is little work in the field of recommendation system, and only a few research works combine these two topics. HyperRec [38] uses the advantages of HGCN to recommend the next item for users. DHCN [39] models the session data as a hypergraph and then extracts the feature information of the session by using the dual-channel hypergraph convolution network, so as to infer the next item in the session. SHARE [40] is different from DHCN in that it uses the hypergraph attention network (HGAT) [31], which can flexibly aggregate the context information of related items in the session to generate item embedding. However, these recommendation methods do not make use of social relations, resulting in unsatisfactory recommendation results. Therefore, we integrate social networks into the recommendation system and exploit the potential information of users by using the characteristics of a hypergraph that can capture complex high-order relations.

## 3. Proposed Method

### 3.1. Preliminaries

#### 3.1.1. Notation Definition

Let *U* = {*u*_1_, *u*_2_, *u*_3_,…, *u*_*m*_} denote a set of *m* users, and let *I* = {*i*_1_, *i*_2_, *i*_3_,…, *i*_*n*_} denote a set of *n* items. We define the user-item interaction matrix *Z* ∈ ℝ^*m*×*n*^ according to the set of items purchased by the user. Elements of *Z* are set to 1 for items purchased by the user and 0 for items that the user has not purchased. In this paper, the social network is undirected, and the friends between users are mutual, so we use *S* ∈ ℝ^*m*×*m*^ to represent the symmetric relation matrix. In the neural network, let *h*_*u*_^(*l*)^ ∈ ℝ^*d*^(*l*)^^ represent the vector representation of user *u* with dimension *d*^*l*^ at layer *l*. In the model, H^(*l*)^ ∈ ℝ^*m*×*d*^(*l*)^^ and P^(*l*)^ ∈ ℝ^*d*^(*l*)^^ are used to represent the embedding vectors of all users and items, respectively. The mathematical notations used in this paper are summarized in Table 1.

#### 3.1.2. Hypergraph Definition

A hypergraph is defined as a graph *G*=(*V*, *E*), where *V*={*v*_1_, *v*_2_, *v*_3_,…, *v*_*N*_} denotes the node set of *N* nodes in the graph, and *E* = {*e*_1_,*e*_2_,*e*_3_,…,*e*_*M*_} denotes the edge set of *M* edges in the graph. The definition of hypergraph *G* is as follows:

(1) $$\begin{array}{c} C_{ij}=\left\{\begin{array}{cc} 1, & \text{if }v_{i}\in e_{j},\\ 0, & \text{if }v_{i}\notin e_{j}. \end{array}\right. \end{array}$$

In equation (1), the incidence matrix *C* ∈ ℝ^*N*×*M*^ represents the topological structure of hypergraph *G*. If the node *v*_*i*_ ∈ *e*_*j*_, the input of the matrix is 1; otherwise, the input is 0.

Generally speaking, the attribute of each node in a hypergraph can be expressed as *X*=[*x*_1_, *x*_2_, *x*_3_,…,*x*_*N*_]^*T*^ ∈ *ℝ*^*N*×*d*^, where *d* refers to the dimension of the node attribute vector.

Compared with simple graphs with degree 2, a hyperedge of a hypergraph can connect multiple nodes, which enhances the correlation of high-order data and breaks through the limitation that simple graphs must be connected in pairs. As shown in Figure 2, the adjacency matrix of the hypergraph is represented by the relation between nodes and hyperedges. Compared with the adjacency matrix composed of nodes in the simple graph, the adjacency matrix greatly alleviates the sparseness of the data and improves the computational efficiency.

In the following section, we present our model HASRE, which represents the application of hypergraph attention network to social recommendation system. In Figure 3, The overall framework diagram of our model is shown.

### 3.2. Hypergraph Construction

In order to better represent the high-order relation between users, we first align the social network graph with the user-item interaction graph and then construct a hypergraph, which includes user nodes, item nodes, and the relation between them. In this paper, we build a hypergraph that uses a triangle structure to represent three semantic topics (as shown in Figure 1). These three semantic themes are the “social theme” of “having the same friends,” “joint theme” of “friends buying the same items,” and “buying theme” of “strangers buying the same items”.

### 3.3. Hypergraph Attention Network

In this paper, the hypergraph channel is mainly used to deal with three types of triangular semantic topics and then extract more accurate user embedding vectors from high-order relations between users. Therefore, it is unreasonable to directly take the basic user embedding vector *H*^(0)^ as input. To control the flow of basic user embedding vectors into different channels, we use a self-gating unit (SGU) [41] filter to filter the input information, specifically defined as

(2) $$\begin{array}{c} H_{c}^{\left(0\right)}=f_{\text{gate}}^{c}\left(H^{\left(0\right)}\right)=H^{\left(0\right)}⊙\sigma \left(H^{\left(0\right)}W_{g}^{c}+b_{g}^{c}\right). \end{array}$$

In equation (2), *W*_*g*_^*c*^ ∈ ℝ^*d*×*d*^ and *b*_*g*_^*c*^ ∈ ℝ^*d*^, respectively, represent the weight parameter and the bias parameter that can be trained in SGU, *c* ∈ {*t*, *r*} represents two different channels, *H*_*t*_^(0)^ refers to the basic user embedding vector for hypergraph channels, *H*_*r*_^(0)^ refers to the basic user embedding vector for explicit social networks, ⊙ represents dot product, and *σ*(.) is the Sigmoid function. SGU adjusts basic user embedding in feature granularity by dimension reweighting and finally obtains user embedding for the hypergraph channel.

Inspired by [37], we use HyperGAT to model the hypergraph constructed in this paper. HyperGAT uses two different aggregation functions to learn the representation of user nodes. Firstly, the feature information of the nodes is aggregated to the hyperedge, and then, the information is aggregated from the hyperedge to the node. These two processes are called node-level attention mechanism and hyperedge-level attention mechanism, respectively.

#### 3.3.1. Node-Level Attention Mechanism

Given a node *v*_*i*_, we first learn the hyperedge representation that connects it through HyperGAT. Because the contribution values of nodes in the hyperedge *e*_*j*_ to the hyperedge are different, the attention mechanism is used to highlight those nodes that are important to the hyperedge. Then, these nodes are aggregated to obtain the representation of hyperedge:

(3) $$\begin{array}{c} f_{j}^{l}=\sigma \left(\sum_{v_{k}\in e_{j}}a_{jk}W_{1}x_{k}^{l-1}\right). \end{array}$$

In equation (3), *σ*(.) is a Sigmoid function, *W*_1_ is a trainable weight matrix, and *x*_*k*_^*l*^ refers to the characteristic information of node *k* in the *l-*th layer neural network.

The feature information of the node X^(0)^ in the hypergraph uses a multilayer perceptron (MLP) [42] to combine the user basic embedding vector H_*t*_^(0)^ and the item basic embedding vector P_*t*_^(0)^ in the hypergraph, as follows:

(4) $$\begin{array}{c} X^{\left(0\right)}=g\left(H_{t}^{\left(0\right)}⊕P_{t}^{\left(0\right)}\right). \end{array}$$

In equation (4), *g* indicates the fusion of user information and item information, ⊕ indicates the series operation between the two vectors, *P*_*t*_^(0)^ is the basic embedded vector of the item in the hypergraph, and the acquisition method is the same as *H*_*t*_^(0)^.

*a*_*jk*_ represents the attention coefficient contributed to the hyperedge when the information of node *k* is aggregated to the hyperedge *e*_*j*_, and its calculation formula is as follows:

(5) $$\begin{array}{c} a_{jk}=\frac{\exp\left(a_{1}^{T}u_{k}\right)}{\sum_{v_{p}\in e_{j}}\exp\left(a_{1}^{T}u_{p}\right)}. \end{array}$$

(6) $$\begin{array}{c} u_{k}=\text{LeakyReLU}\left(W_{1}x_{k}^{l-1}\right).\; \end{array}$$

In equations (5) and (6), *a*_1_^*T*^ is the weight parameter, and *u*_*k*_ refers to the correlation degree of node *k* on the hyperedge *e*_*j*_.

#### 3.3.2. Hyperedge-Level Attention Mechanism

All hyperedges are represented by {*f*_*j*_^*l*^*|*∀ *e*_*j*_ ∈ *E*_*i*_}. The hypergraph structure designed in this paper is mainly used to learn accurate user embedding vectors by using the high-order relation between users. If the node *v*_*i*_ in the hypergraph is a user node, we use the hyperedge information to learn the node information of the next layer of users. The specific calculation formula is as follows:

(7) $$\begin{array}{c} h_{i}^{l}=\;\sigma \left(\sum_{e_{j}\in E_{i}}b_{ij}W_{2}f_{j}^{l}\right). \end{array}$$

In equation (7), *h*_*i*_^*l*^ is the updated feature information of node *v*_*i*_, *W*_2_ represents the weight matrix, and *b*_*ij*_ refers to the attention coefficient of hyperedge *e*_*j*_ on node *v*_*i*_, which can be calculated by the following formula:

(8) $$\begin{array}{c} b_{ij}=\frac{\exp\left(a_{2}^{T}v_{j}\right)}{\sum_{e_{p}\in E_{i}}\exp\left(a_{2}^{T}v_{p}\right)}, \end{array}$$

(9) $$\begin{array}{c} v_{j}=\text{LeakyReLU}\left(\left[\left.W_{2}f_{j}^{l}\right\|W_{1}h_{i}^{l-1}\right]\right). \end{array}$$

In equation (8) and equation (9), *a*_2_^*T*^ is the weight parameter, *v*_*j*_ refers to the correlation of the hyperedge *e*_*j*_ at node *i*, and || is the connection operation of the vector.

The hypergraph includes user nodes and item nodes. Through the attention mechanism at the node level, the hyperedge information of the hypergraph can be obtained. Because the hypergraph structure designed in this paper is mainly to use the high-order relation between users to learn accurate user embedding vectors, item information only plays an auxiliary role in the hypergraph. Therefore, if the node *v*_*i*_ of the hypergraph is a user node, the hyperedge information is aggregated to the user node by using the attention mechanism at the hyperedge level. Finally, we can get the user's potential feature vector *H*_*t*_^(*l*)^ from *l-*th Layer HyperGAT.

### 3.4. Learning Comprehensive User Representations and Item Representations

After user embedding propagated through the L-layer HyperGAT, we average the user embedding obtained by each layer in the hypergraph channel to form the final user representation for the hypergraph channel:

(10) $$\begin{array}{c} H_{t}=\frac{1}{L+1}\sum_{l=0}^{L}H_{t}^{\left(l\right)}. \end{array}$$

In equation (10), *H*_*t*_ represents the user embedding vector obtained after averaging *L* layer HyperGAT propagation, and *H*_*t*_^(*l*)^ refers to the user's potential feature vector obtained from the *l* layer HyperGAT.

The social relations of users are complex. Paying attention to the high-order social relations defined by us in hypergraph, there are some isolated users in social networks. Therefore, we use a simple graph convolution neural network to extract user feature vectors and item feature vectors in a user-item interaction graph.

(11) $$\begin{array}{c} H_{r}^{\left(l+1\right)}=D_{u}^{-1}ZP^{\left(l\right)},\;H_{r}^{\left(0\right)}=f_{\text{gate}}^{r}\left(H^{\left(0\right)}\right), \end{array}$$

(12) $$\begin{array}{c} \begin{array}{c} P^{\left(l+1\right)}=D_{i}^{-1}Z^{T}H_{m}^{\left(l\right)},\\ H_{m}^{\left(l\right)}=\frac{1}{2}H_{t}^{\left(l\right)}+\frac{1}{2}H_{r}^{\left(l\right)}. \end{array} \end{array}$$

In equation (11) and equation (12), *H*_*r*_^(*l*)^ is the gated user embedding of graph convolution channel, *H*_*m*_^*l*^ is the combination of the user embedding of hypergraph channel and the user embedding of graph convolution channel, and *D*_*u*_ ∈ ℝ^*m*×*m*^ and *D*_*i*_ ∈ ℝ^*n*×*n*^ are the degree matrices of *Z* and *Z*^T^, so that the final user embedding vector *H* and item embedding vector *P* can be obtained:

(13) $$\begin{array}{c} \begin{array}{c} H=H_{t}+\frac{1}{L+1}\sum_{l=0}^{L}H_{r}^{\left(l\right)},\;\\ P=\frac{1}{L+1}\sum_{l=0}^{L}P^{\left(l\right)}. \end{array} \end{array}$$

Equation (13) shows that after propagating through *L* layers of neural networks, we obtain the final user embedding vector *H* and item embedding vector *P* by averaging neural networks of each layer.

### 3.5. Model Optimization

In order to learn the model parameters of HASRE, we need an objective function to optimize our model. For implicit feedback from users, we use Bayesian Personalized Ranking (BPR) loss for training.

(14) $$\begin{array}{c} {ℒ}_{BPR}=\sum_{i\in I\left(u\right),j\notin I\left(u\right)}-\log\;\sigma \left({\hat{r}}_{u,i}\left(\Phi \right)-{\hat{r}}_{u,j}\left(\Phi \right)\right)+\lambda {\left\|\Phi \right\|}_{2}^{2}.\; \end{array}$$

In equation (14), Φ is the parameter of HASRE, ${\hat{r}}_{u,i}$ refers to the predicted score of user *u* on item *i*, and *σ*(.) refers to the Sigmoid function. To reduce the generalized error, the *L*_2_-regularization method with superparameter *λ* is used here. In addition, to optimize the objective function of this model, we use small batch Adam as the optimizer in actual operation. Its main advantage is that it calculates the adaptive learning rate simultaneously of training, which reduces the pain of choosing the appropriate learning rate, thus ensuring stability at the beginning of training without preheating.

### 3.6. Complexity Analysis

Here, we analyze the complexity of the computational cost of the model in this paper. The computational cost of the HASRE model is mainly composed of a hypergraph attention network, graph convolution network, and self-gating mechanism. For the hypergraph attention network passing through *L* layers, the propagation consumption is less than *O*(*N*‖*M|dL*), where *N* is the number of nodes in the hypergraph and *M* is the number of hyperedges in the hypergraph. Similarly, the time complexity of a graph convolution network is *O*(|*Z*^+^|*dL*), where *Z* represents the number of nonzero elements in |*Z*^+^|. For the self-gating mechanism, each gating unit contains (*d*+1) × *d* parameters, so its time complexity is *O*(*md*^2^). From the overall analysis, the total complexity of our model is *O*(|*N*‖*M*|*dL*+|*Z*^+^|*dL*+*md*^2^).

## 4. Experiment

### 4.1. Dataset

We used three public datasets related to the recommendation system, LastFM, Douban, and Yelp, to evaluate all the models, Table 2 summarizes the specific information of these data sets.

1. LastFM : LastFM dataset contains the user's social network, tags, and information about the music artists that each user listens to frequently
2. Douban: Douban data set is a data set about Douban movies crawled by community netizens. The data includes social relations between users, ratings, and comments of users on movies, basic information about movies, and basic information about actors
3. Yelp: Yelp data set is a business information data set, which is used for personal, educational, and academic purposes. This data includes Yelp business, users' comments on enterprises, and users' social networks

### 4.2. Baselines

To evaluate the recommended performance of this model, we compare HASRE with the following baseline methods.

1. BPR [43]: BPR is the basic model of all implicit feedback recommendation methods.
2. SBPR [44]: SBPR uses social relations as a more accurate ranking-based model, by assuming that users tend to assign higher rankings to items that their friends prefer.
3. LightGCN [45]: LightGCN processes the internal structure of GCN and uses GCN with only neighbor aggregation structure for collaborative filtering, which is more suitable for recommendation system.
4. GraphRec [46]: GraphRec is a social recommendation algorithm based on a graph neural network. Its main purpose is to integrate social relations into the recommendation system and realize user-item and user-user interaction.
5. DiffNet++ [10]: DiffNet++ is an improvement of the DiffNet algorithm, which models the diffusion of friends' influence and users' interest in a unified framework.
6. DHCF [47]: DHCF is a new recommendation method based on hypergraph, which uses hypergraph to model high-order correlation information.

In order to evaluate the recommendation performance of this model, we will compare it with the above six representative models. These representative models include the recommendation system BPR without a social network, the traditional social recommendation system SBPR, the social recommendation system LightGCN, GraphRec, and DiffNet++ based on GNNs, and the emerging recommendation system DHCF based on hypergraph neural network.

### 4.3. Evaluation Metric

To evaluate the performance of all the recommended models, *Precision@K*, *Recall@K*, and *NDCG@K* are experimentally calculated. Among them, *Precision@K* refers to the proportion of the top-*K* items that each user likes in the recommended system. *Recall@K* refers to the proportion of related items in the top-*K* recommendations of each user. When the *K* value is fixed, the accuracy is only determined by true positive samples, while the recall rate is determined by both true positive and false positive samples. NDCG is used as an evaluation index for ranking results, considering the order of ranking lists under ideal conditions. *Precision* is defined as

(15) $$\begin{array}{c} \text{Precision}@K=\frac{\sum_{i=1}^{K}rel_{i}}{\min\left(K,\left|y_{u}^{rec}\right|\right)}. \end{array}$$

In equation (15), *rel*_*i*_=1/0 indicates whether the item ranked *i* in the top*-K* recommendation list appears in the test set, and *y*_*u*_^*rec*^ indicates the number of items rated by user *u* in the recommendation list. *Recall* is defined as

(16) $$\begin{array}{c} \begin{array}{c} \text{Recall}@K=\frac{\sum_{i=1}^{K}rel_{i}}{\min\left(K,\left|y_{u}^{\text{test}}\right|\right)} \end{array}. \end{array}$$

In equation (16), *rel*_*i*_=1/0 indicates whether the item ranked *i* in the top-*K* recommended lists appears in the test set, and *y*_*u*_^test^ indicates the number of items scored by user *u* in the test set. *NDCG* is defined as

(17) $$\begin{array}{c} NDCG@K=\frac{DC\;G@K}{I\;DC\;G@K}. \end{array}$$

In equation (17), *DCG@K* and *IDCG@K* are

(18) $$\begin{array}{c} DCG@K=\sum_{i=1}^{K}\frac{2^{rel_{i}}-1}{\log_{2}\left(i+1\right)}, \end{array}$$

(19) $$\begin{array}{c} IDCG@K=\sum_{i=1}^{\left|REL\right|}\frac{2^{rel_{i}}-1}{\log_{2}\left(i+1\right)}. \end{array}$$

In equation (18) and equation (19), *rel*_*i*_ indicates the hierarchical correlation at the *i*-th position, and |*REL*| indicates that the collection is composed of the top-*K* according to the order of correlation from large to small.

The higher the values of *Precision@K*, *Recall@K*, and *NDCG@K*, the better the performance. We evaluate each ranking list with *K* = 10 (as shown in Table 3).

### 4.4. Experimental Settings

The experimental operating system is Linux, using Python version 3.6, based on TensorFlow version 1.14 to achieve this model, and benefits from GPU to accelerate the training process of the model.

We randomly use 80% of user-item interaction data as a training set to learn parameters, 10% of the data as the verification set to adjust parameters, and finally 10% of the data as the test set to compare performance. The codes of the comparison methods used in this paper are all from Github, the parameters are all specified in the author's paper, and the experimental results are obtained on the data set in this paper. For the sake of fairness, the hyperparameters of all models are set as follows: the learning rate is 0.001, the potential embedded dimension d is set to 50, the iteration is 100 times, the batch size is 2000, the regularization coefficient *λ* = 0.001, and the model is optimized by Adam. We describe the influence of different parameters (*d*, *λ*, and the depth) of HASRE in Section 4.7, and we use the best parameter settings in Section 4.5 and Section 4.6.

### 4.5. Recommendation Performance

In this paper, LastFM, Douban and Yelp data sets are used for experimental analysis, and the experimental results of system performance comparison are shown in Table 3.

In traditional recommendation systems, recommendation system that uses social network information usually performs better than those that do not use social network information. For example, SBPR performs better than BPR on all data sets. The recommendation system based on GNNs is better than the traditional recommendation system. In the social recommendation system, the recommendation performance of GraphRec and DiffNet++ is obviously better than that of SBPR, especially the average index of DiffNet on LastFM, Douban, and Yelp data sets improved by 1.898%, 1.709%, and 0.564%, respectively, compared with SBPR. In the general recommendation, compared with BPR, LightGCN has the most obvious comparison on the LastFM data set, and *P@10*, *R@10*, and *N@10* have improved by 3.599%, 3.659%, and 3.176%, respectively. The performance of these models is to be expected. On the one hand, because social network information plays an auxiliary role in general recommendation system and complements the interactive information of historical items, it can help users learn their preferences well; on the other hand, because GNNs can model social network graphs and user-item interaction graph, taking into account the importance of neighbor nodes in the graph, it can greatly improve the accuracy of recommendation system.

In the recommendation system based on GNNs, the general recommendation system LightGCN has better recommendation performance than the social recommendation system GraphRec and DiffNet++. This can be attributed to the simplification of GCN by the LightGCN model. Because GCN is modified on the basis of a convolution neural network, it contains a variety of neural network operations. LightGCN abandons the feature transformation and nonlinear activation function of GCN and only applies neighbor aggregation to cooperative filtering. However, GrphRec and DiffNet++ may be limited by these useless neural networks, resulting in lower recommended performance than LightGCN.

The supergraph structure model has better expression ability than the graph structure model in theory, while DHCF based on HGCN does not show good recommendation performance compared with other recommendation systems based on graph convolution neural network LightGCN and DiffNet++. The poor performance of the DHCF model is probably due to the inapplicability of the hyperedge construction method of the model, which leads to the high density of the matrix. The overall performance of the model HASRE proposed in this paper is better than other recommendation system models on the three data sets (the optimal value is shown in bold). Taking LastFM data as an example, compared with the traditional recommended method SBPR with the best performance, HASRE improved by 3.376%, 3.516%, and 3.868% on P @ 10, *R* @ 10, and N @ 10, respectively. Compared with DiffNet++, which is the best social recommendation method based on graph neural networks, HASRE improves by 1.382%, 1.482%, and 1.774% on *P@10*, *R@10,* and *N@10*, respectively. Combined with the above analysis, there are two main factors for the good performance of HASRE. First, the auxiliary role of social network information on the recommendation system. Secondly, HyperGAT can capture complex high-order user relations and fully consider the different influences of different neighbors of user nodes in the hypergraph.

### 4.6. Ablation Study

In order to verify that each component in the model has a positive contribution to the model proposed in this paper, we carried out ablation experiments and compared HASRE and its three variants (experimental results are shown in Figure 4).

1. UISRE: We remove the hypergraph attention network from HASRE, and the user embedding vector is the basic user embedding vector. The extraction of the item embedding vector is consistent with that described in this model, which is extracted from the user-item interaction graph through a graph convolution network
2. GASRE: GASRE is a variant of HASRE removing hypergraph structure, which uses graph attention network to generate user embedding in the traditional social graph
3. HCSRE: We replace hypergraph attention network with hypergraph convolution neural network, so as to extract user embedding vector from hypergraph

As shown in Figure 4, from the experimental results of the comparison model, UISRE obtained the worst results. Although it uses GCN to extract the feature vectors of items, it does not take into account the relation between users. Based on the UISRE model, GASRE adopted graph structure and GAT to consider the simple pairwise user relation on the social graph. The recommendation performance of this model is better than UISRE, indicating that it is necessary to model the relation between users based on the graph structure. Next, to model the high-order relations of users by using hypergraph structure, we construct the same hypergraph according to the same process as HASRE, but in HCSRE, we use HCNN to aggregate user information from adjacent hyperedges, which can improve the accuracy of recommendations better than using the traditional social graph. This shows the effectiveness of hypergraph structure and the importance of modeling high-order relations for users. However, it still lags behind HASRE, because it does not fully consider the different effects of node information and hyperedge information on user nodes.

### 4.7. Parameter Sensitivity Analysis

In this paper, we construct multiple HyperGAT layers to model the information flow between users with high-order connections in a hypergraph, which can be regarded as high-order information propagation. We overlay the hypergraph attention network layer from 1 layer to 5 layers. As shown in Figure 5, HASRE achieves optimal performance when the number of layers of the hypergraph attention network is 2. When the hypergraph attention network layers are stacked to more than 2 layers, the performance of HASRE on all data is degraded. The analysis of the above results shows that the shallow structure is more suitable for HASRE. With the increase of HyperGAT layers, the performance of HASRE decreases, probably because the hypergraph attention network learns the data so thoroughly that it also learns the characteristics of noise data [48].

Through the above analysis, when the hypergraph attention network is 2 layers, the model achieves the best recommendation effect. On this basis, we analyze the embedding dimension *d* and the regularization coefficient *λ* of the model. We set the change of *d* to {10, 30, 50, 80, 100}, and Figure 6 shows how the performance metric *Precision@*10 varies over the three datasets in this paper with different *d* values. In general, with the increase of embedding dimension, the performance of the model will increase at first and then decrease. When we increase the embedding dimension from 10 to 50, we can significantly improve the performance. However, when the embedded dimension exceeds 50, the model performance will show a downward trend. The research shows that the smaller embedding dimension may decrease the performance of the model, while too larger embedding dimension may lead to overfitting of the model. At the same time, we set the change of *λ* to {0, 0.0005, 0.001, 0.005, 0.01}, so as to analyze its impact on the performance of the model. As shown in Figure 7, when *λ* = 0.001, the model obtains the best performance. Therefore, we can draw a conclusion that an appropriate *λ* value can effectively prevent the occurrence of overfitting and underfitting.

## 5. Conclusion

This paper proposes a model that applies the hypergraph attention network to the social recommendation system (HASRE), which improves the performance of the recommendation system to some extent. Specifically, the HASRE model uses a hypergraph structure to capture the high-order relations between users, which makes up for the defect of the traditional graph structure that can only connect pairs of user nodes. In addition, to fully consider the different influences of users' friends on them, we integrate graph attention networks into hypergraph structure and assign more appropriate weights to each user's neighbors, which greatly improves the performance of the model. The performance of this model is verified on three real data sets. From their test results, the model has certain advantages and can indeed improve the accuracy of recommendations.

In this paper, we only use social networks in the recommendation system, and the actual application also contains a lot of attribute information of items. Therefore, exploring social recommendations system with attribute information will also be an interesting research direction. In addition, social information is dynamic in real life, and the model only considers static social information. In the future, we will consider applying dynamic graph neural networks to social recommendation systems to better mine users' potential preferences, which is expected to further improve the performance of recommendation systems.

## Figures and Tables

**Figure 1:** Three common semantic theme motifs for high-order user relations in social recommendation systems.

**Figure 2:** Hypergraph network structure.

**Figure 3:** The Model Framework of applying hypergraph attention network to social recommendation system (HASRE).

**Figure 4:** Ablation experimental results.

**Figure 5:** The influence of the number of HyperGAT layers on HASRE.

**Figure 6:** Effect of embedding size on datasets.

**Figure 7:** Impact of *λ* in *L*_2_-regularization.

**Table 1:** Summary of notations.

Symbol	Definitions and descriptions
*U*	User set
*I*	Item set
*V*	Point set of hypergraph
*E*	Edge set of hypergraph
*d*	The size of the embedding vector
*X*	The embedding vector of hypergraph nodes
*Z*	The user-item interaction matrix
*S*	The social relation matrix
*H* ^(*l*)^	The embedding vector representation of all users in the l-th layer
*P* ^(*l*)^	The embedding vector representation of all items in the l-th layer
*H*_*t*_^(*l*)^	The basic user embedding vector for hypergraph channels
*H*_*r*_^(0)^	The basic user embedding vector for explicit social networks
*W*	The weight in neural network
*b*	The bias in neural network
⊕	The concatenation operator of two vectors

**Table 2:** Dataset statistics.

Location	#User	#Item	#Interactions	#Relations
Lastm	1892	17632	92834	25434
Douban	2848	39586	894887	35770
Delicious	19539	21266	450884	363672

**Table 3:** Comparative experimental results of recommendation system performance.

Method	LastFM			Douban			Yelp		
	P@10 (%)	R@10 (%)	N@10 (%)	P@10 (%)	R@10 (%)	N@10 (%)	P@10 (%)	R@10 (%)	N@10 (%)
BPR	15.606	15.821	18.953	15.673	5.160	17.476	2.002	5.173	3.840
SBPR	16.491	16.703	20.216	15.993	5.322	17.821	2.192	5.468	4.314
DHCF	16.877	17.131	20.744	16.871	5.755	18.655	2.298	5.986	4.700
GraphRec	17.385	18.020	21.173	17.021	5.916	19.051	2.323	6.075	4.653
DiffNet	18.485	18.737	22.310	17.532	6.205	19.701	2.480	6.354	4.833
LightGCN	19.205	19.480	23.392	17.780	6.247	19.881	2.586	6.525	4.998
HASRE	**19.867**	**20.219**	**24.084**	**18.817**	**6.982**	**21.699**	**2.865**	**7.122**	**5.691**

## Data Availability

We used three public datasets in this paper, LastFM, Douban, and Yelp. The LastFM dataset can be obtained from http://files.grouplens.org/datasets/hetrec2011. The Douban dataset comes from the website https://pan.baidu.com/s/1hrJP6rq. The Yelp dataset can be obtained from https://www.dropbox.com/sh/h97ymblxt80txq5/AABfSLXcTu0Beib4r8P5I5sNa?dl=0.
